The article "Metaheuristics with Deep Learning-Enabled Parkinson's Disease Diagnosis and Classification Model" was published in 2022. Journal: J Healthc Eng.

# Metaheuristics with Deep Learning-Enabled Parkinson's Disease Diagnosis and Classification Model

**DOI:** 10.1155/2022/9276579

**Published:** 2022-01-10

**Authors:** Adel A. Bahaddad, Mahmoud Ragab, Ehab Bahaudien Ashary, Eied M. Khalil

**Affiliations:** ^1^Information Systems Department, Faculty of Computing and Information Technology, King Abdulaziz University, Jeddah 21589, Saudi Arabia; ^2^Information Technology Department, Faculty of Computing and Information Technology, King Abdulaziz University, Jeddah 21589, Saudi Arabia; ^3^Centre of Artificial Intelligence for Precision Medicines, King Abdulaziz University, Jeddah 21589, Saudi Arabia; ^4^Mathematics Department, Faculty of Science, Al-Azhar University, Nasr City 11884, Cairo, Egypt; ^5^Electrical and Computer Engineering Department, Faculty of Engineering, King Abdulaziz University, Jeddah 21589, Saudi Arabia; ^6^Mathematics Department, College of Science, Taif University, Taif 21944, Saudi Arabia

## Abstract

Parkinson's disease (PD) affects the movement of people, including the differences in writing skill, speech, tremor, and stiffness in muscles. It is significant to detect the PD at the initial stages so that the person can live a peaceful life for a longer time period. The serious levels of PD are highly risky as the patients get progressive stiffness, which results in the inability of standing or walking. Earlier studies have focused on the detection of PD effectively using voice and speech exams and writing exams. In this aspect, this study presents an improved sailfish optimization algorithm with deep learning (ISFO-DL) model for PD diagnosis and classification. The presented ISFO-DL technique uses the ISFO algorithm and DL model to determine PD and thereby enhances the survival rate of the person. The presented ISFO is a metaheuristic algorithm, which is inspired by a group of hunting sailfish to determine the optimum solution to the problem. Primarily, the ISFO algorithm is applied to derive an optimal subset of features with a fitness function of maximum classification accuracy. At the same time, the rat swarm optimizer (RSO) with the bidirectional gated recurrent unit (BiGRU) is employed as a classifier to determine the existence of PD. The performance validation of the IFSO-DL model takes place using a benchmark Parkinson's dataset, and the results are inspected under several dimensions. The experimental results highlighted the enhanced classification performance of the ISFO-DL technique, and therefore, the proposed model can be employed for the earlier identification of PD.

## 1. Introduction

Parkinson's disease (PD) is a brain disorder that occurs as a consequence of the loss of brain cells. It mainly affects body mobility. Its symptom gradually becomes evident. Some of these symptoms that perform at early stages are tremors, slowness in movement, poor body posture, rigidness in muscles, deviation in speech, handwriting strokes, and imbalance [1]. In this disorder, a person's nerve cell gradually loses their ability to communicate between them, which results in nervous system disorders such as depression. This disease must be diagnosed at earlier stages because it is incurable. When the accurate symptom of PD is recognized with their relative weightage, then doctors can suggest a pathology lab test for this feature and diagnosis might take place at an initial consultation itself. It will result in an earlier diagnosis of Parkinson's disease. The symptoms such as changes in speaking patterns and handwriting strokes might assist in an earlier diagnosis of this disorder [2]. Erdogu Sakar and team lately received a speech dataset by examining the pronunciation of vowels “a” and “o” of disease-affected persons. Except speaking patterns, handwriting stroke patterns might help in detecting the disorder [3]. Factors studied for distinguishing a person from a healthier patient are individual age, fare handedness (right/left), maximum and mean distance among given summary in test, handwriting strokes noted in the drawing, and test time duration.

Recently, data have been improved by number of instances and numbers of features that make data noisier [4]. The noisier datasets could create the model to decrease the predicted accuracy, increase the computation cost, increase the complexity, and train the data slower. Therefore, feature selection developed an essential task for machine learning (ML) beforehand training the models [5]. The feature selection (FS), also known as attribute selection, is a method that focuses on finding a subset from the provided comprehensive set of features and fewer downgrades of the system performance; thus, the subsets of feature forecast the target with accuracy analogous to the performances of the original set of features and with the reducing computation costs. The FS method is categorized into wrapper-based and filter-based algorithms. The filter-based method utilizes a statistical method for finding the vital of all features (attributes). The wrapper-based method utilizes the machine-learning (ML) method. The wrapper-based method is computationally costly when compared to the filter-based method [6]. The wrapper method is additionally classified as heuristic search algorithm and sequential search algorithm.

An evolutionary algorithm is a part of artificial intelligence (AI) system that primarily focused on biological evolution. Biological evolution includes 4 major procedures such as selection, reproduction, mutation, and recombination [7]. Different from conventional optimization models, evolutionary algorithms depend on random sampling. This process is continuously employed on the solution officially reported as population, and the FF was employed for determining the quality of solutions. This solution changes based on the evolutionary procedure that finally assists to discover the global solution to the problems [8]. The evolutionary method has been recognized for performing well under distinct scenarios since it does not consider the fundamental fitness landscape. Even an easy evolutionary algorithm could easily resolve difficult challenges [9]. The only drawbacks in the evolutionary algorithm are the computational cost factor that is decreased by the fitness function calculation.

This study presents an improved sailfish optimization algorithm with deep learning (ISFO-DL) model for PD diagnosis and classification. The presented ISFO-DL technique designs an ISFO-based feature selection technique to derive an optimal subset of features with a fitness function of maximum classification accuracy. At the same time, the rat swarm optimizer (RSO) with the bidirectional gated recurrent unit (BiGRU) is employed as a classifier to determine the existence of PD. The experimental validation of the IFSO-DL model is carried out using a benchmark Parkinson's dataset, and the results are inspected under several dimensions.

The rest of the paper is arranged as follows.  Section 2 offers the related works, Section 3 provides the proposed model, Section 4 inspects the performance validation, and Section 5 draws the conclusion.

## 2. Related Works

Huseyn [10] presented the DL methodology for realizing healthy people, analysis of PD, and multiple system atrophy. Oh et al. [11] employed the EEG signal of 20 PD and 20 standard subjects in this work. A 13-layer CNN framework could conquer the requirement for the traditional feature representation phases that are carried out. Wang et al. [12] introduced a novel deep-learning model for the earlier detection and classification of PD using the premotor features. In particular, to diagnose PD at earlier stages, various symptoms have been taken into account. Shahid and Singh [13] developed a DNN method with the decreased input feature space of Parkinson's telemonitoring datasets for predicting PD evolution. PD is a progressive and chronic nervous system disorder, which impacts the motion of body. PD is measured by utilizing the unified PD rating scale (UPDRS).

Kaur et al. [14] surged a feasible medical decision-making method, which assists the medical professionals in detecting the PD-affected person. In this study, a certain architecture-based grid searching optimization method is presented for developing an enhanced DL algorithm to forecast the earlier diagnosis of PD; therefore, various hyperparameters are to be tuned and set for the assessment of DL algorithm. The grid searching optimization method includes its performance, the optimization of DL method, and the hyperparameters. In the study by Sivaranjini S. and Sujatha [15], an effort has been made for classifying the MR images of healthier control and PD subjects with the DL-NN model. The CNN framework AlexNet is utilized for refining the detection of PD. The MR image is tested to provide the accuracy measures and trained with the transfer learned network.

Quan et al. [16] presented a Bi-LSTM method for capturing the time-series dynamic feature of a speech signal to PD diagnosis. The dynamic speech feature is evaluated on the basis of energy content evaluation from the transition under voiced to unvoiced segments (offset) and the transition from unvoiced to voiced segments (onset). Sigcha et al. [17] proposed a novel methodology-based RNN and a single waist-worn triaxial accelerometer for enhancing the FOG recognition accuracy to be utilized in real home environment.

Leung et al. [18] focused on developing DL, an ensemble method for the prediction in person with PD. The initial and next phases of the method extracted features from DaTscan and medical measures of motor symptoms, respectively. Then, an ensemble of DNN model was trained on distinct subsets of the extracted feature for predicting the person results from 4 years afterward early baseline screening. Masud et al. [19] introduced an ACSA- and DL-based optimal FS technique. The presented method is the integration of CROW Search and DL (CROWD) SSAE-NN. PD dataset has been taken for experimental purposes.

## 3. The Proposed ISFO-DL Model

In this study, the ISFO-DL technique has been developed for PD detection and classification. The proposed ISFO-DL technique is mainly intended to determine PD and thereby enhance the survival rate of the person. The presented ISF-DL technique involves three major processes namely ISFO-based feature selection, BiGRU-based classification, and RSO-based hyperparameter optimization. These three processes are elaborated in the succeeding sections.

### 3.1. Design of ISFO-Based Feature Selection Technique

At this stage, the ISFO algorithm is employed to choose an optimal subset of features and thereby boost the classifier results. Research has established that group hunting is the major social behavior in groups of fish, birds, mammals, and arthropods. In comparison with individual hunting, group hunting could save the energy utilization of the hunter to attain the aim of catching prey. Sailfish is employed for saving the present optimum solution, although sardines are applied in the searching space for finding an optimal solution. The arithmetical expression of the model is given as follows.

The population locations of sardines and sailfish are arbitrarily initiated, and every sardine and sailfish are allocated a randomized location *X*_*SF*(*i*)_^*k*^ and *X*_*S*  *D*(*j*)_^*k*^, successively, where *i* ∈ {sail  fish}, *j* ∈ {sardlines}, and *k* represent the iteration count. The upgraded location of sailfish has been arithmetically given as follows:

(1) $$\begin{array}{c} X_{SF\left(i\right)}^{k+1}=X_{\mathrm{eliie}}^{k}-\mu_{k}\times \left(\mathrm{rand}\left(0,1\right)\times \frac{X_{\mathrm{elite}}^{k}+X_{\mathrm{injure}}^{k}}{2}-X_{SF\left(i\right)}^{k}\right)\;, \end{array}$$

(2) $$\begin{array}{c} \mu_{k}=2\times \mathrm{rand}\left(0,1\right)\times \mathrm{Pd}-\mathrm{Pd,} \end{array}$$

(3) $$\begin{array}{c} \mathrm{Pd=1}-\frac{\mathrm{NumSP}}{\mathrm{NumSF+NumSD}}. \end{array}$$

Let *X*_*SF*(*i*)_^*k*^ be the preceding location of the ith sailfish, and *μ*_*k*_ indicates a coefficient created at kth iteration, using equation (2). To conserve the optimum solution of all the iterations, the sardine and sailfish with optimal fitness value are known as “elite” sailfish and “injured” sardine, respectively, and their location at iteration *k* is represented as *X*_eilie_^*k*^ and *X*_injure_^*k*^.*P*  *d* denotes the density of prey sardines that indicates the number of prey in all the iterations, as in equation (3). NumSF and NumSD stand for the population of sailfish and sardines [20], and the relation is NumSP=NumSD× percent, in which percent characterizes the primary species of sailfish as a percentage of sardine populations.

A novel location of the sardines at *k* iteration is estimated as follows:

(4) $$\begin{array}{c} X_{S\;D\left(j\right)}^{k+1}=\mathrm{rand}\left(0,1\right)\times \left(X_{\mathrm{elite}}^{k}-X_{S\;D\left(j\right)}^{k}+\mathrm{ATK}\right), \end{array}$$

(5) $$\begin{array}{c} \mathrm{ATK}=A\times \left(1-\left(2\times \mathrm{iter}\times \varepsilon \right)\right), \end{array}$$

(6) $$\begin{array}{c} \alpha =\mathrm{NumSD\times ATK}, \end{array}$$

(7) $$\begin{array}{c} \beta =d\times \mathrm{ATK}. \end{array}$$

Here, *X*_*S*  *D*(*j*)_^*k*^ signifies the preceding location of the *jth* sardine. iter denotes the amount of existing iterations. ATK means the sailfish attacking strength, i.e., decreased linearly on all the iterations given by equation (5). Once the *A*=4 and *ε*=0.001, if ATK < 0.5, the amount of sardines that upgrade the location (*α*) and the number of parameters of them (*β*) is evaluated by equations (6) and (7). When ATK ≥ 0.5, each sardine gets upgraded.

For simulating the procedure of the sailfish catching sardines, when *f*(SD_*j*_) < *f*(SF_*i*_), then the location of later can be substituted with the place of the sardine *i*, as follows:

(8) $$\begin{array}{c} X_{\mathrm{SF}\left(i\right)}^{k}=X_{S\;D\left(j\right)}^{k}\;f\left(SD_{j}\right)<f\left(SF_{i}\right). \end{array}$$

Chaotic mapping algorithms have both randomness and certainty and stochastic behavior and nonlinear motion. Chaos concept is the study of dynamic systems. The stimulating property of this system is that if there is a slight modification in the algorithm, the entire algorithm gets affected. The research has shown that the primary value of chaotic technique, the population of metaheuristic model, was initiated based on the relationship of chaotic mapping, and chaotic order was made, which could efficiently save the variety of populations and conquer the premature problems of traditional optimization method.  Figure 1 illustrates the process flow of SFO technique.

The population initiation of sardines and sailfish in the SFO is a stochastic approach. It is based on population initiation while searching for an optimum solution. For enhancing the global searching capacity of the model and preventing the problems that the diversities of sardine and sailfish population reduce in late searches, hence we proposed a population initialization of sailfish and sardines using tent chaotic operator. The tent map can be described as follows:

(9) $$\begin{array}{c} T_{i+1}=\left\{\begin{array}{cc} \frac{T_{i}}{0.7}, & T_{i}\leq 0.7,\\ \frac{1-T_{i}}{0.3}, & T_{i}>0.7. \end{array}\right.. \end{array}$$

In the equation, *T*_*i*_ denotes that the sequence of ith iteration (*T*_*i*_ ∈ (0,1))  indicates the tent chaotic sequence distribution of *T*_*n*_ with the primary value *T*_0_=0.9 in 200 iterations. Next, the sardine and sailfish populations are initiated:

(10) $$\begin{array}{c} X_{\mathrm{SF}\left(i+1\right)}=T_{i+1}\times \left(X_{\mathrm{ub}}-X_{\mathrm{lb}}\right)+X_{\mathrm{lb}}\;,\\ X_{\text{SD}\left(j+1\right)}=T_{j+1}\times \left(X_{\mathrm{ub}}-X_{\mathrm{lb}}\right)+X_{\mathrm{lb}}. \end{array}$$

While *X*_*SF*(*i*+1)_ and *X*_*S*  *D*(*j*+1)_ indicate the location value of individual sardines and sailfish, *X*_ub_ and *X*_lb_ represent the upper and lower bounds of the individual sardines and sailfish in each dimension.

Assume the novel feature set be ℱ={*f*_1_, *f*_2_,   …, *f*_*D*_}, where *D* implies the entire amount of features or dimension of feature set, and consider the class label be *C*={*c*_1_,   …,  *c*_*l*_}, where *l* stands for the amount of classes. The FS technique determines a subset *S*={*s*_1_,   …,  *s*_*m*_}, where *m* < *D*, *S* ⊂ ℱ, and *S* is minimal classification error rate than some other subsets of similar size or some appropriate subset of *S*. FS is the binary optimized issue, where the solution was restricted to binary values from 0 to 1. At this point, the solution has signified utilizing a binary vector where 1 refers that the equivalent feature was chosen and 0 demonstrates the equivalent feature is not chosen. The size of this vector was equivalent to the number of features from the original dataset. The ISFO was presented for solving continuous optimized issues in which the solution contains the real value. For mapping the continuous search space of typical ISFO to binary one, it can utilize a transfer function [21]. It can be utilized as a sigmoid transfer function and written as follows:

(11) $$\begin{array}{c} T\left(x\right)=\frac{1}{1+e^{-x}}. \end{array}$$

At this point, utilizing the probability value attained in equation (11), the present place of sailfish was upgraded by the following equation:

(12) $$\begin{array}{c} X^{d}\left(t\right)=\left\{\begin{array}{cc} 1, & \mathrm{if}\;\mathrm{rnd}<T\left(X^{d}\left(t\right)\right),\\ 0, & \mathrm{if}\;\mathrm{rnd}\geq T\left(X^{d}\left(t\right)\right). \end{array}\right.. \end{array}$$

Usually, the FS is a multiobjective issue, with 2 objectives: (a) for achieving maximum classification accuracy (for instance, maximized issue) and (b) for selecting minimal number of features (for instance, minimized issue). Using equation (15), these 2 objectives are joined and the FS issue was changed to single-objective issue.

(13) $$\begin{array}{c} ↓\mathrm{Fitness}\;=\omega \gamma \left(S\right)+\left(1-\omega \right)\frac{\left|S\right|}{D}, \end{array}$$

where *S* stands for the chosen feature subset, |*S*| defines the cardinality of chosen feature subset or the number of chosen features, *γ*(*S*) signifies the classification error rate of *S*, *D* refers the novel dimensional of dataset, and *ω* ∈ [0,1] signifies weight.

### 3.2. Design of the RSO-BiGRU-Based Classification Model

During the classification process, the RSO-BiGRU model is applied to carry out the classification process. Learning is a continuous representation that is effective to control sequential data. An RNN is mostly appropriate to encoded sequential data.  Figure 2 demonstrates the framework of BiGRU. During this analysis, it can utilize BiGRU for learning [22]. The computation of BiGRU was separated into 2 parts: forward and reverse order data broadcasts. To provide sentence *X*=(*x*_1_,  *x*_2_,   …, *x*_*n*_), *x* ∈ ℝ^*k*^, *x* refers the concatenating vector of present word and place, and the forward GRU was computed as follows:

(14) $$\begin{array}{c} i=\sigma \left(W_{xi}x_{t}+W_{hi}h_{t-1}+b_{i}\right), \end{array}$$

(15) $$\begin{array}{c} f=\sigma \left(W_{xf}x_{t}+W_{hf}h_{t-1}+b_{f}\right), \end{array}$$

(16) $$\begin{array}{c} g=\tanh\left(W_{xg}x_{t}+W_{hg}\left(i⊙h_{t-1}\right)+b_{g}\right), \end{array}$$

(17) $$\begin{array}{c} h_{t}=\left(1-f\right)⊙h_{t-1}+f⊙g, \end{array}$$

where *W*_*∗*_ and *b*_*∗*_ signify the weight matrix and bias vectors, respectively; *σ* refers the sigmoid functions; and ⊙ stands for the element-wise multiplication. *x*_*t*_ implies the input word vector at time steps *τ*, and *h*_*t*_ signifies the hidden state of current time step *r*.$\vec{h_{i}}$ and $\overset{\leftarrow }{h_{i}}$ demonstrate the outcome of forward and backward GRUs, respectively. The BiGRU output is represented as follows:

(18) $$\begin{array}{c} h_{i}^{\mathrm{bi-gru}}=\left[\vec{h_{i}};\overset{\leftarrow }{h_{i}}\right]. \end{array}$$

To effectively tune the hyperparameters involved in the BiGRU model, the RSO is applied to it.

The rats are territory animals that live from the set of combined males and females. The performance of rats is very aggressive from several analyses that are outcome from the death of any animals. This aggressive performance is a vital simulation of this work but chase and fight with prey. The chasing and fighting behavior of the rats can be used to model the RSO algorithm and can be utilized to solve optimization problems. This subsection explains the performance of rats, for instance, chasing and fighting. Afterward, the presented RSO technique is summary.

#### 3.2.1. Chasing the Prey

In general, the rats are social animals to chase the prey under the set with situation social agonistic efficiency. For defining this efficiency mathematically, it can be assumed that optimum search agents have skill of place of the prey. Another search agent has upgraded its places in terms of optimum search agents attained so far. The subsequent formulas are presented under this process:

(19) $$\begin{array}{c} \vec{P}=A\cdot {\vec{P}}_{i}\left(x\right)+C\cdot \left({\vec{P}}_{r}\left(x\right)-{\vec{P}}_{i}\left(x\right)\right), \end{array}$$

where ${\vec{P}}_{i}\left(x\right)$ demonstrates the places of rats and ${\vec{P}}_{r}\left(x\right)$ signifies the better optimum solutions.

However, *A* and *C* parameters were calculated as follows:

(20) $$\begin{array}{c} A=R-x\times \left(\frac{R}{\mathrm{Ma}x_{\mathrm{Iteration}}}\right)\mathrm{where},\;x=0,1,2,\;\ldots ,\;\mathrm{Ma}x_{\mathrm{Iteration}}, \end{array}$$

(21) $$\begin{array}{c} C=2\cdot \mathrm{rand}\left(\right)\text{.} \end{array}$$

So, *R* and *C* imply the arbitrary numbers among [1, 5] and [0,2], respectively. The parameters *A* and *C* are responsible for optimum exploration and exploitation over the course of rounds.

#### 3.2.2. Fighting with Prey

For mathematically defining the fight procedure of rats with prey, the subsequent formula was projected:

(22) $$\begin{array}{c} {\vec{P}}_{i}\left(x+1\right)=\left|{\vec{P}}_{r}\left(x\right)-\vec{P}\right|, \end{array}$$

where ${\vec{P}}_{i}\left(x+1\right)$ implies the upgraded next places of rat. It stores the optimum solution and upgrades the places of other search agents in terms of optimum search agent. The rat (*A*,  *B*) upgraded their place nearby the place of prey (*A*^*∗*^, *B*^*∗*^). By altering the parameters as revealed in equations (20) and (21), the distinct amount of places is achieved on the present place [23]. Also, this technique is comprehensive from *n*-dimensional environments. Consequently, the exploration and exploitation have been guaranteed using the value of parameters *A* and *C*. The projected RSO technique stores optimum solutions with many operators.

## 4. Performance Validation

This section inspects the PD classification result analysis of the presented IFSO-DL technique. The results are investigated against four datasets namely HandPD Spiral, HandPD Meander, Speech PD, and Voice PD [24–26].  Table 1 and Figure 3 offer the selected features attained by the IFSO-DL technique with other FS methods. The results show that the IFSO-DL technique has chosen the least number of features compared with other FS techniques on all test datasets. For instance, with the HandPD Spiral dataset with 13 features, the IFSO-DL technique has selected a set of 4 features, whereas the MGOA, MGWO, and OCFA techniques have chosen a total of 5, 7, and 8 features, respectively.

Likewise, with the HandPD Meander dataset with 13 features, the IFSO-DL system has selected a set of 6 features, whereas the MGOA, MGWO, and OCFA methods have chosen a total of 8, 8, and 7 features, respectively. Meanwhile, with the Speech PD dataset with 23 features, the IFSO-DL system has selected a set of 10 features, whereas the MGOA, MGWO, and OCFA techniques have chosen a total of 11, 12, and 13 features, respectively. Eventually, with the Voice PD dataset with 26 features, the IFSO-DL manner has selected a set of 7 features, whereas the MGOA, MGWO, and OCFA algorithms have chosen a total of 8, 9, and 17 features, respectively.

Table 2 offers a detailed comparative result analysis of the IFSO-DL technique with recent methods on the test HandPD Spiral dataset. The results show that the MGWO-KNN and MGOA-KNN techniques have obtained lower accuracy of 0.734 and 0.756, respectively. In line with this, the MGOA-DT technique has attained moderate accuracy of 0.890. At the same time, MGOA-RF, MGWO-RF, and MGWO-DT techniques have accomplished reasonable accuracy of 0.929, 0.924, and 0.924, respectively. However, the IFSO-DL technique has outperformed the other techniques with the maximum accuracy, DR, and FAR of 0.933, 0.982, and 0.080, respectively.

Figure 4 demonstrates the accuracy of graph analysis of the IFSO-DL technique on the test HandPD Spiral dataset. The figure portrays that the IFSO-DL technique has gained increased training and validation accuracies. It is noted that the IFSO-DL technique has accomplished improved validation accuracy over the training accuracy.

The loss graph analysis of the IFSO-DL technique is investigated in Figure 5. The figure shows that the IFSO-DL technique has accomplished enhanced outcomes with the lower validation loss compared with training loss. It also demonstrates that the IFSO-DL technique has obtained reduced validation loss compared with training loss.

Table 3 suggests a detailed comparative outcome analysis of the IFSO-DL technique with recent approaches on the test HandPD Meander dataset. The results outperformed that the MGWO-KNN and MGOA-KNN systems have obtained minimum accuracy of 0.728 and 0.748, respectively. Afterward, the MGOA-DT manner has gained moderate accuracy of 0.890. Also, MGOA-RF, MGWO-RF, and MGWO-DT systems have accomplished reasonable accuracy of 0.937, 0.930, and 0.880, respectively. However, the IFSO-DL method has exhibited the other methodologies with the maximal accuracy, DR, and FAR of 0.940, 1.000, and 0.135, respectively.

Figure 6 reveals the accuracy graph analysis of the IFSO-DL manner on the test HandPD Meander dataset. The figure shows that the IFSO-DL technique has reached improved training and validation accuracies. It can be clear that the IFSO-DL algorithm has accomplished improved validation accuracy over the training accuracy.

The loss graph analysis of the IFSO-DL system is studied in Figure 7. The figure portrays that the IFSO-DL technique has accomplished enhanced outcomes with the lower validation loss related to training loss. It also outperforms that the IFSO-DL technique has gained lower validation loss related to training loss.

Table 4 provides a brief comparative outcome analysis of the IFSO-DL system with recent approaches on the test Speech PD dataset. The results depicted that the MGWO-KNN and MGOA-KNN methods have obtained minimal accuracy of 0.918 and 0.897, respectively. Besides, the MGOA-DT technique has reached moderate accuracy of 0.846. Likewise, MGOA-RF, MGWO-RF, and MGWO-DT methods have accomplished reasonable accuracy of 0.949, 0.939, and 0.898, respectively. However, the IFSO-DL technique has shown the other algorithms with the maximal accuracy, DR, and FAR of 0.953, 1.000, and 0.185, respectively.

Figure 8 displays the accuracy graph analysis of the IFSO-DL approach on the test Speech PD dataset. The figure demonstrates that the IFSO-DL technique has achieved higher training and validation accuracies. It can be obvious that the IFSO-DL technique has accomplished increased validation accuracy over the training accuracy.

The loss graph analysis of the IFSO-DL algorithm is explored in Figure 9. The figure depicts that the IFSO-DL technique has accomplished superior results with the lower validation loss compared with training loss. It can also portray that the IFSO-DL technique has reached reduced validation loss related to training loss.

Table 5 provides a detailed comparative outcome analysis of the IFSO-DL manner with recent techniques on the test Voice PD dataset. The results demonstrated that the MGWO-KNN and MGOA-KNN methodologies have gained minimal accuracy of 0.858 and 0.918, respectively. Similarly, the MGOA-DT technique has achieved moderate accuracy of 1.000. Subsequently, MGOA-RF, MGWO-RF, and MGWO-DT methods have accomplished reasonable accuracy of 1.000, 1.000, and 1.000, respectively. Finally, the IFSO-DL technique has displayed the other algorithms with the higher accuracy, DR, and FAR of 1.000, 1.000, and 0.000, respectively.

Figure 10 exhibits the accuracy graph analysis of the IFSO-DL system on the test Voice PD dataset. The figure portrays that the IFSO-DL technique has reached increased training and validation accuracies. It is noticeable that the IFSO-DL methodology has accomplished higher validation accuracy over the training accuracy.

The loss graph analysis of the IFSO-DL approach is examined in Figure 11. The figure outperforms that the IFSO-DL method has accomplished enhanced outcomes with the lesser validation loss related to training loss. It also shows that the IFSO-DL manner has obtained reduced validation loss connected to training loss.

Figure 12 shows the accuracy analysis of the IFSO-DL technique with other recent techniques on the four test datasets [27]. The figure portrays that the IFSO-DL technique has gained effective outcomes with the maximum accuracy values on all the test datasets.

Figure 13 illustrates the DR analysis of the IFSO-DL algorithm with other recent manners on the four test datasets. The figure shows that the IFSO-DL technique has achieved effective outcomes with the maximal DR values on all the test datasets.

Figure 14 depicts the FAR analysis of the IFSO-DL method with other recent approaches on the four test datasets. The figure outperforms that the IFSO-DL system has reached effective outcomes with higher FAR values on all the test datasets. From the abovementioned tables and figures, it is apparent that the IFSO-DL technique has been found to be an effective tool for PD detection and classification.

## 5. Conclusion

In this study, the ISFO-DL technique has been developed for PD detection and classification. The proposed ISFO-DL technique is mainly intended to determine PD and thereby enhance the survival rate of the person. The presented ISF-DL technique involves three major processes namely ISFO-based feature selection, BiGRU-based classification, and RSO-based hyperparameter optimization. The design of ISFO and RSO algorithms finds useful to significantly enhance the PD classification performance. The experimental validation of the IFSO-DL model is carried out using a benchmark Parkinson's dataset, and the results are inspected under several dimensions. The experimental results highlighted the enhanced classification performance of the ISFO-DL technique, and therefore, the proposed model can be employed for the earlier identification of PD. In future, the PD classification performance can be boosted by the use of outlier detection and clustering approaches.

## Figures and Tables

**Figure 1:** Process flow of SFO.

**Figure 2:** Structure of BiGRU.

**Figure 3:** FS analysis of the IFSO-DL technique with 4 datasets.

**Figure 4:** Accuracy analysis of IFSO-DL technique under the HandPD Spiral dataset.

**Figure 5:** Loss analysis of IFSO-DL technique under the HandPD Spiral dataset.

**Figure 6:** Accuracy analysis of IFSO-DL technique under the HandPD Meander dataset.

**Figure 7:** Accuracy analysis of IFSO-DL technique under the HandPD Meander dataset.

**Figure 8:** Accuracy analysis of IFSO-DL technique under the Speech PD dataset.

**Figure 9:** Loss analysis of IFSO-DL technique under the Speech PD dataset.

**Figure 10:** Accuracy analysis of IFSO-DL technique under the Voice PD dataset.

**Figure 11:** Loss analysis of IFSO-DL technique under the Voice PD dataset.

**Figure 12:** Accuracy analysis of IFSO-DL technique with existing approaches.

**Figure 13:** DR analysis of IFSO-DL technique with existing approaches.

**Figure 14:** FAR analysis of IFSO-DL technique with existing approaches.

**Table 1:** Selected features of existing with the proposed model.

Dataset	Total features	MGOA	MGWO	OCFA	IFSO-DL
HandPD Spiral	13	5	7	8	4
HandPD Meander	13	8	8	7	6
Speech PD	23	11	12	13	10
Voice PD	26	8	9	17	7

**Table 2:** Result analysis of existing with the proposed IFSO-DL model on the HandPD Spiral dataset.

Methods	Accuracy	DR	FAR
MGOA-KNN	0.756	0.853	0.531
MGOA-RF	0.929	0.979	0.219
MGOA-DT	0.890	0.947	0.281
MGWO-KNN	0.734	0.819	0.500
MGWO-RF	0.924	0.940	0.119
MGWO-DT	0.924	0.940	0.119
IFSO-DL	0.933	0.982	0.080

**Table 3:** Result analysis of existing with the proposed IFSO-DL model on the HandPD Meander dataset.

Methods	Accuracy	DR	FAR
MGOA-KNN	0.748	0.858	0.476
MGOA-RF	0.937	1.000	0.191
MGOA-DT	0.890	0.918	0.167
MGWO-KNN	0.728	0.858	0.600
MGWO-RF	0.930	0.991	0.222
MGWO-DT	0.880	0.920	0.222
IFSO-DL	0.940	1.000	0.135

**Table 4:** Result analysis of existing with the proposed IFSO-DL model on the Speech PD dataset.

Methods	Accuracy	DR	FAR
MGOA-KNN	0.897	0.967	0.300
MGOA-RF	0.949	1.000	0.222
MGOA-DT	0.846	0.900	0.300
MGWO-KNN	0.918	0.974	0.300
MGWO-RF	0.939	1.000	0.300
MGWO-DT	0.898	0.949	0.300
IFSO-DL	0.953	1.000	0.185

**Table 5:** Result analysis of existing with the proposed IFSO-DL model on the Voice PD dataset.

Methods	Accuracy	DR	FAR
MGOA-KNN	0.918	0.835	0.009
MGOA-RF	1.000	1.000	0.000
MGOA-DT	1.000	1.000	0.000
MGWO-KNN	0.858	0.803	0.081
MGWO-RF	1.000	1.000	0.000
MGWO-DT	1.000	1.000	0.000
IFSO-DL	1.000	1.000	0.000

## Data Availability

The dataset used in this study is publicly available via the following link: https://wwwp.fc.unesp.br/∼papa/pub/datasets/Handpd/.
